This article has been retracted.

# Hypoxia-inducible factor 1a induces phenotype switch of human aortic vascular smooth muscle cell through PI3K/AKT/AEG-1 signaling

**DOI:** 10.18632/oncotarget.16448

**Published:** 2017-03-22

**Authors:** Kai Liu, Changcun Fang, Yuwen Shen, Zhengqin Liu, Min Zhang, Bingbing Ma, Xinyan Pang

**Affiliations:** ^1^ Department of Cardiovascular Surgery, Qilu Hospital of Shandong University, Jinan 250012, Shandong, China

**Keywords:** HIF-1a, HASMC, PI3K/AKT/AEG-1

## Abstract

To date, hypoxia-inducible factor 1a (HIF-1a) and astrocyte elevated gene-1 (AEG-1) have been involved in the proliferation, migration and morphological changes of vascular smooth muscle cells. However, the potential relationship of HIF-1a-AEG-1 pathway in human aortic smooth muscle cell (HASMC) has not been reported. In the present study, in-vitro assays were utilized to explore the potential impact of HIF-1a-AEG-1 signaling on HASMC phenotype. Here, we found that HIF-1a expression was up-regulated in the media of thoracic aortic dissection tissues as compared with normal aortic tissues, and was associated with increased apoptotic SMCs and decreased AEG-1 expression. Mechanically, hypoxia promoted the expression of HIF-1a by PI3K-AKT pathway in HASMCs; HIF-1a further suppressed the expressions of AEG-1, a-SMA and SM22a, and promoted osteopontin (OPN) expression. Functionally, HIF-1a inhibited the proliferation and migration of HASMCs. However, si-HIF-1a or Akt inhibitor abrogated HIF-1a-mediated related expressions and biological effects above. In conclusion, HIF-1a induces HASMC phenotype switch, and closely related to PI3K/AKT and AEG-1 signaling, which may provide new avenues for the prevention and treatment of aortic dissection diseases.

## INTRODUCTION

As is known to all, vascular smooth muscle cells (VSMCs) act as a key member in the media of human aorta, which have two kinds of cell phenotypes, including contractile and synthetic status. Contractile VSMCs have a poor capacity of proliferation and migration, and showed a spindle-like model. Notably, contractile VSMCs were very hard to generate extracellular matrix [1–4]. Synthetic VSMCs have a stronger ability of proliferation, migration and synthesis of extracellular matrix, including collagen, elastin, and proteoglycans [4, 5]. It has reported that the biomarkers of contractile VSMC involve smooth muscle α-actin (α-SMA) and smooth muscle 22α (SM22α), and the biomarkers of synthetic VSMC involve osteopontin (OPN) [5–7]. In some cardiovascular events, like atherosclerosis, hypertension, and aortic dissection, contractile VSMCs are able to change into synthetic VSMCs, which could trigger the migration, proliferation and synthesis of extracellular matrix of VSMCs [5, 6, 8, 9]. In recent years, some extracellular factors and downstream signaling are implicated into this switch of VSMCs [4, 5, 8, 10–12].

HIF-1α has been reported as a hypoxia-inducible nuclear factor in VSMCs, which plays important roles in hypoxic response of mammalian cells, and is able to modulate hypoxia-inducible genes [13]. Additionally, HIF-1α can bind to hypoxia-inducible genes to regulate cell biology, which included inducible nitric oxide synthase, VEGF, and the glycolytic enzymes aldolase A, enolase 1, lactate dehydrogenase A, and phosphoglycerate kinase 1 [14, 15]. Besides, PI3K/AKT is recommended as a crucial signaling that controls the phenotype of VSMCs [15]. The specific regulation effects of PI3K/AKT on VSMC phenotype and biology depends on different stimuli or some unknown downstream transcription factors [16]. In our previous study, AEG-1 was also identified as an important factor that regulates muscle cell growth, proliferation and differentiation. Although AEG-1 may be involved in VSMC phenotypic switch, its specific role and its relationship with HIF-1/PI3K/AKT signaling are not clear.

We assumed that HIF-1α can be induced by PI3K/AKT signaling pathway to regulate alteration of AEG-1 expression in human aortic VSMCs, leading to phenotype switch of HASMCs. In the present study, the *in-vitro* experiments including RT-PCR and western blot were utilized to explore the potential impact of HIF-1α-AEG-1 signaling on SMC cell phenotype.

## RESULTS

### HIF-1α expression in aortic SMCs of TAD specimens

In the present study, we used qRT-PCR and western blot to analyze the expression of HIF-1α in aortic SMCs of thoracic aortic dissection (TAD) specimens. Our data revealed that the expression level of HIF-1α mRNA and protein in the aortic media of TAD tissues showed an increase by 3.5 and 3.2 respectively as compared with the normal aortic tissues (Figure 1). Besides, the expression level of HIF-1α mRNA and protein in other aortic structures of TAD tissues showed no significant changes as compared with the same structures of normal aortic tissues (Figure 1). These findings identified that HIF-1α expression is significantly increased in aortic SMCs of TAD specimens.

**Figure 1:** HIF-1α expression is upregulated in media of TAD specimens The expression of HIF-1α mRNA and protein in TAD and normal tissues was detected by RT-PCR **(A)** and western blot **(B)**, and was normalized to that of GAPDH mRNA and protein, respectively. **(C)** Each dot represents the relative expression level of HIF-1α mRNA and protein of tissue samples (n=30 for TAD, n=12 for normal tissues) with the line indicating the mean level; *P <0.01 by paired t test.

### HIF-1α expression is positively associated with the rate of apoptotic SMCs

It has been reported that apoptosis can account for the loss of SMCs of aortic media. To explore the effects of HIF-1α on cell apoptosis of aortic SMCs, we investigated the association between HIF-1α expression and the apoptotic rate of aortic SMCs. We found that few TUNEL-positive cells can be detected in normal control aortic tissues. However, the number of TUNEL-positive cells showed a significant increase in the media of TAD tissues. Statistically, we also found that the expression of HIF-1α is positively associated with the rate of TUNEL-positive cells in TAD tissues (Figure 2).

**Figure 2:** HIF-1α expression is positively associated with the rate of apoptotic SMCs **(A)** The percentage of TUNEL positive cells was significantly higher in TAD than that in normal tissues. Red arrow indicates TUNEL positive cells, bar =50 μm; *P <0.01 by paired t test. **(B)** Dot plots represent log10 percentage of apoptotic cells against log10 HIF-1α protein expression level. The lines represent approximated curves. The correlation coefficient (r) and the P value indicate the statistical significance of the positive correlation between the x and y variables.

### AEG-1 expression is negatively associated with the expression of HIF-1α in aortic media of TAD tissues

AEG-1 expression can be demonstrated to be increased in some proliferative cells. In our previous study, we also demonstrated the role of AEG-1 in the development of cardiac muscle cells. Consistent with the previous studies, western blot assay identified that the expression of AEG-1 in aortic media of TAD tissues became significantly decreased compared with that in normal aortic tissues (Figure 3A). To further elucidate the potential association between AEG-1 and HIF-1α expression, we conducted the correlation analysis using western blot data, and found that expression of AEG-1 was obviously negatively associated with the expression of HIF-1α in TAD tissues (Figure 3B), indicating that HIF-1α is likely to down-regulate the expression of AEG-1 in aortic SMCs of TAD specimens.

**Figure 3:** AEG-1 expression is negatively associated with the expression of HIF-1α in aortic media of AD tissues **(A)** Representative images of AEG-1 bands in aortic media of TAD and normal tissues. Expression level of AEG-1 protein was significantly higher in TAD than in normal. **(B)** Dot plots represent log10 AEG-1 expression against log10 HIF-1α protein expression level. The lines represent approximated curves. The correlation coefficient (r) and the P value indicate the statistical significance of the negative correlation between the x and y variables.

### Hypoxia induces HIF-1α expression in aortic SMCs

In *in-vitro* assay, we exposed human aortic VSM cells to 1% of oxygen to induce the expression of HIF-1α. We found that the expression of HIF-1α mRNA started to arise at the first 4 h (about 4.0-fold), and then peaked at 8 h (6.0-fold). Afterwards, the expression of HIF-1α mRNA showed a significant decrease at 24 h (Figure 4A). By contrast, the level of HIF-1α expression shows no significant increase in normal oxygen group. Induction of HIF-1α expression by hypoxia in cultured human aortic VSM cells seems to be consistent with its expression in the media of TAD tissues. As expected, the expression of HIF-1α mRNA in cultured VSM cells is obviously associated with increased HIF-1α protein levels (Figure 4B).

**Figure 4:** Hypoxia induces HIF-1α expression in aortic SMCs In in-vitro assay, we exposed human aortic VSM cells to 1% of oxygen to induce the expression of HIF-1α. HIF-1α mRNA and protein were detected using RT-PCR **(A)** and western blot assay **(B)**. GAPDH was used as a loading control. The intensity of bands was quantified using image J software and normalized to GAPDH. Data shown are means ± SEM of at least three independent experiments. *p<0.001, using one-way ANOVA.

### HIF-1α induces apoptosis of aortic SMCs

To investigate the effect of HIF-1α on cell apoptosis of human aortic SMCs, the apoptosis of human aortic SMCs transfected with HIF-1α plasmids was assayed using flow cytometry. We observed that the expression of HIF-1α mRNA and protein was obviously increased in the aortic SMCs with HIF-1α plasmids as compared with vectors at post-infection 48 h (Figure 5). Subsequently, we conducted annexin V-FITC assay, and found the rate of annexin V-FITC+/PI- plus annexin V-FITC+/PI+ in aortic SMC cells with HIF-1α plasmids were significantly increased than that in control cells (Figure 5B). These results suggested that overexpression of HIF-1α facilitates the apoptosis of human aortic SMCs.

**Figure 5:** HIF-1α induces apoptosis of aortic SMCs **(A)** Aortic SMCs were infected with HIF-1α plasmids (or vectors) at a MOI of 100. The expression of HIF-1α and its effect on cell apoptosis were detected at 72 hr post-infection. The expression level of HIF-1α mRNA and protein was detected by qRT-PCR and western blot and normalized to that of GAPDH. **(B)** Cells were stained with annexin V-FITC and propidium iodide (PI). Flow cytometric contour plots showed the percentage of stained cells. Histogram showed the percentage of Annexin V+/PI- and Annexin V+/PI+ cells of HIF-1α-infected and vector-infected aortic SMCs.

### HIF-1α affects proliferations and migrations in human aortic SMCs

Based on results above, we continued to conduct the CCK-8 assay, and found that the OD value of human aortic SMCs transfected with HIF-1α plasmids was significantly decreased as compared with vector control group, and their differences were significant statistically (P<0.01) (Figure 6A). This finding suggested that HIF-1α plasmids significantly affect the proliferations of HA-VSMCs. Besides, we carried out the transwell assay, and found that the numbers of migrating cells in human aortic SMCs transfected with HIF-1α plasmids was significantly decreased as compared with vector control group, and their differences were significant statistically (P<0.01) (Figure 6B). This finding suggested that HIF-1α plasmids significantly affect the migration of HA-VSMCs.

**Figure 6:** HIF-1α affects proliferations and migrations in human aortic SMCs **(A)** Comparison of the OD value in the different groups with CCK-8 test (The resulting data were represented as x¯±SD, *P<0.01 vs. Blank control group). **(B)** Comparison of the number of migrating cells in the different groups with transwell migration assay. (The resulting data were represented as x¯±SD, *P<0.01 vs. Blank control group).

### HIF-1α promotes phenotype switch of aortic SMCs

To explore the effect of HIF-1α on the phenotypic switch of aortic SMCs, RT-PCR and western blotting were used to detect the expression of α-SMA, and the rate of α-SMA-positive cells was assayed using flow cytometry in human aortic SMCs transfected with HIF-1α plasmids. As shown in Figure 7A-7B, we demonstrated that the expression of α-SMA mRNA and protein was obviously decreased in HIF-1α plasmids-treated SMCs cells than vector-treated cells. Additionally, the rate of α-SMA-positive SMCs transfected with HIF-1α plasmids was also significantly decreased compared with that in vector-treated SMCs (Figure 7C). Based on the molecular level, the expression of OPN in HIF-1α plasmids group was significantly increased, while the expression of SM22α was obviously decreased as compared with vector control. These differences were statistically significant (P<0.01) (Figure 7A-7B). HIF-1α induces the expression of OPN and suppresses the expression of α-SMA and SM22α in human aortic VSMCs. These data indicates that HIF-1α plasmids indeed change the phenotype of aortic SMCs from contractile phenotype to synthetic phenotype.

**Figure 7:** HIF-1α promotes phenotype switch of aortic SMCs To explore the effect of HIF-1α on the phenotypic switch of aortic SMCs, RT-PCR **(A)** and western blotting **(B)** were used to detect the expression, and the rate of α-SMA **(A)**/SM22α **(B)**-positive cells was assayed using flow cytometry **(C)** in human aortic SMCs transfected with HIF-1α plasmids.

### Hypoxia induces PI3K, P-PI3K, AKT, P-AKT and suppressed AEG-1 by HIF-1α

The PI3K, p-PI3K, AKT, and p-AKT levels in hypoxia group was increased, while their levels in normal oxygen group were decreased; these differences were significant statistically (P<0.01). However, AEG-1 level in hypoxia group was decreased, while its level in normal oxygen group were increased; these differences were significant statistically (P<0.01) (Figure 8A). Afterwards, in the hypoxia group, Akt inhibitor suppressed hypoxia-induced increase of OPN and HIF-1α protein levels, while Akt inhibitor attenuated the expression of α-SMA, SM22α and AEG-1 proteins. Besides, the PI3K and P-PI3K levels in hypoxia-AKT inhibitor group showed no statistically significant differences with hypoxia-control group. In addition, Akt inhibitor exhibited the similar effects with DMSO control in the normoxia group (Figure 8B). To further identify this pathway, we used si-HIF-1α to transfect aortic SMCs, and found that si-HIF-1α suppressed hypoxia-induced increase of OPN and HIF-1α protein levels, and promoted the expression of α-SMA, SM22α and AEG-1 in the hypoxia group. Besides, the PI3K, P-PI3K, AKT, P-AKT levels showed no statistically significant differences with si-control group in the hypoxia group. As expected, si-HIF-1α exhibited the similar effects with si-control in the normoxia group (Figure 8B). (Figure 8C). These findings indicated that hypoxia induced PI3K, p-PI3K, AKT, and p-AKT expressions, and further activated the expression of HIF-1α, leading to suppression of AEG-1 expression and SMC phenotype switch.

**Figure 8:** Hypoxia induces PI3K, p-PI3K, AKT, p-AKT and suppressed AEG-1 by HIF-1α In this work, SMCs were subjected to different conditions, including **(A)** (hypoxia, normoxia), **(B)** (hypoxia: Akt inhibition, hypoxia: DMSO; normoxia: Akt inhibition, normoxia: DMSO), and **(C)** (hypoxia: si-HIF-1α, hypoxia: si-control; normoxia: si-HIF-1α, normoxia: si-control). The relative expressions levels of various proteins in the different groups with western blotting.

## DISCUSSION

To date, the pathogenesis of TAD have been investigated widely, and increasing evidence showed that some factors were involved in the pathogenesis of TAD, including patient heredity like Marfan syndrome, hypertension, atherosclerosis, inflammation and autoimmune disorders [17, 18]. However, the molecular mechanisms underlying the development and progression of TAD are still not elucidated. As is known to all, the normal aortic media comprises of many vascular smooth muscle cells that are regularly arranged and distributed widely, and extracellular matrix that is enriched in elastic fibers. Obviously, SMCs would play an essential role in the development of progression of TAD, which may be involved in the structure and function of aortic tissues [19, 20]. In normal human body, contractile phenotype of VSMCs plays an important role in maintenance of the vascular structure and function of the blood vessel wall. When TAD occurred, the number and rate of synthetic VSMCs are reported to be obviously increased, resulting in decreased aortic elasticity and rupture of blood vessel wall [21–23]. These studies indicated that phenotype switch of SMCs may become a crucial factor implicated into the occurrence of TAD.

More and more studies identified that HIF-1α may be associated with phenotypic switch of VSMCs. Diverse signaling routes are implicated into HIF-1α-induced SMC biology and phenotype switch, including PI3K/AKT signaling pathways. PI3K was demonstrated to be an intracellular signaling molecule, and shares catalytic activities that can activate the downstream molecules. PI3K is able to phosphorylate AKT protein to induce the expression of target genes [24, 25]. As reported, the PI3K/AKT signaling was involved in the regulation of different biological progression, involving cell growth, mitosis and apoptosis. It should be noted that the PI3K/AKT signaling also mediated the regulation of contractile function of vascular smooth muscle, leading to VSMC dysfunction that showed imbalance of vasoconstriction and vascular remodeling [26, 27]. At the same time, some studies also identified that PI3K/AKT regulates the phenotype switch of VSMCs [4]. In addition, our previous study identified that the expression of AEG-1 facilitates the proliferation and migration of SMCs, thus the loss of AEG-1 expression may be an important factor of occurrence of TAD disease. Generally, we assumed that hypoxia-induced HIF-1α participates in phenotypic switch of SMCs probably via PI3K/AKT pathway, and further lead to decreased proliferation and migration via down-regulating the expression of AEG-1.

In the present study, we found that the expression level of HIF-1α mRNA and protein in the aortic media of TAD tissues showed an increase by 2.9 and 2.5 respectively as compared with the normal aortic tissues, and the expression of HIF-1α is positively associated with the rate of TUNEL-positive cells in TAD tissues. In addition, the expression of AEG-1 in aortic media of TAD tissues became significantly decreased than that in normal aortic tissues. We conducted the correlation analysis using western blot data, and found that expression of AEG-1 was obviously negatively associated with the expression of HIF-1α in TAD tissues, indicating that HIF-1α is likely to down-regulate the expression of AEG-1 in aortic SMCs of TAD specimens.

Functionally, we exposed human aortic VSM cells to 1% of oxygen to induce the expression of HIF-1α. To strengthen the expression of HIF-1α, we used HIF-1α plasmids to induce the overexpression of HIF-1α, and observed that overexpression of HIF-1α facilitates the apoptosis and affects proliferations and migrations of human aortic SMCs. Based on molecular level, we found that the expression of OPN in HIF-1α plasmids group was significantly increased, while the expression of α-SMA and SM22α was obviously decreased as compared with vector control. These results suggested that HIF-1α promotes phenotype switch of aortic SMCs. Furthermore, we found that hypoxia induces PI3K, P-PI3K, AKT, P-AKT expressions, indicating that PI3K may directly regulate the expressions of downstream proteins and genes.

Following the introduction of AKT inhibitor, Akt inhibitor suppresses hypoxia-induced increase of OPN and HIF-1α mRNA levels, while Akt inhibitor attenuated the expression of α-SMA, SM22α and AEG-1. To further identify this pathway, we used si-HIF-1α to transfect aortic SMCs, and found that si-HIF-1α suppresses hypoxia-induced increase of OPN and HIF-1α, mRNA levels, and promoted the expression of α-SMA, SM22α and AEG-1. Besides, the PI3K, P-PI3K, AKT, P-AKT levels showed no statistically significant differences with control group. Consistent with Liu et al [28], the activated PI3K/AKT signaling is related to increased levels of some phosphorylated proteins, and inhibitors of PI3K/AKT signaling are able to affect the phosphorylation of downstream proteins. In the present work, we confirmed that hypoxia-induced HIF-1α participates in phenotypic switch of SMCs probably via PI3K/AKT pathway, and further lead to decreased proliferation and migration via down-regulating the expression of AEG-1.

Our studies have a few limitations. Synthetic VSMCs are characterized by secretion of extracellular matrix. However we did not detect the expression levels of collagen, elastin or more extracellular matrix proteins; Thus, it is very hard to identify the role of HIF-1α-AEG-1 in secretion of extracellular matrix. We hope this study needs further exploration. Because the phenotypic switch of VSMCs is associated with occurrence of TAD and many cardiovascular events, thus, investigation of VSMC phenotype switch will be crucial for prevention and treatment of some cardiovascular diseases. In addition, AEG-1 may directly or indirectly affect the expression of biomarkers of phenotype switch, which needs to be identified in the future.

In conclusion, our study identified that the PI3K/AKT and AEG-1 signaling are involved in HIF-1α-induced human aortic VSMCs phenotypic switch. In addition, hypoxia-induced HIF-1α participates in phenotypic switch of SMCs probably via PI3K/AKT pathway, and further lead to decreased proliferation and migration via down-regulating the expression of AEG-1. Thus, the prevention of phenotypic switch may provide new avenues for TAD patients, and more mechanisms need further investigation.

## MATERIALS AND METHODS

### Tissue sampling

Aortic dissection specimens were obtained from 30 patients of acute type A TAD who underwent aortic replacement procedures at Qilu hospital between Jan 2014 and Jan 2016. Aortic tissues from patients with hereditary connective tissue defects, such as Marfan's syndrome, traumatic aneurysms or luetic aortic aneurysms were excluded. Control aortic specimens were obtained from 12 donors. The subjects with TADs and controls showed no significantly difference in clinical features including age, gender, smoking status, hypertension or diabetes. During surgery, full-thickness aortic wall specimens were collected from patients who underwent surgical repair of TAD (ascending aortas above the sinuses of Valsalva). Control specimens from normal ascending aortas were obtained from 12 organ donors. The aortic tissue was carefully cleared of adventitia, and was frozen fresh for Western blot analysis and RT-PCR. The present study was conducted in accordance with the World Medical Association Declaration of Helsinki and was approved by the Medical Ethics Committee of Qilu Hospital. All participants signed informed consents.

### Total RNA extraction and quality test

Total RNA was extracted using TRIzol reagent (Invitrogen; Thermo Fisher Scientific, Inc., Waltham, MA, USA) and purified using the RNeasy mini kit (Qiagen China Co., Ltd., Shanghai, China), according to the manufacturer's instructions. The purity of the total RNA was tested using a NanoDrop 2000 spectrophotometer (Thermo Fisher Scientific, Inc., Wilmington, DE, USA) with 2 μl total RNA per sample, and integrity was tested using an Agilent 2100 BioAnalyzer (Agilent Technologies, Inc., Santa Clara, CA, USA).

### Validation of expression profiles by RT-qPCR

RT-qPCR was performed using the same batch of specimens. The RNAs were extracted using TRIzol reagent, reverse transcribed using Moloney murine leukemia virus (Takara Biotechnology Co., Ltd., Shiga, Japan), and separately subjected to PCR amplification. The primers were synthesized by Invitrogen (Thermo Fisher Scientific, Inc.) using GAPDH as the reference gene. The primer sequences, amplification length and annealing temperature are reported previously [10]. The reaction procedure was as follows: Initial denaturation at 94°C for 5 min; followed by 35 cycles for denaturation at 94°C for 30 sec, annealing for 30 sec and elongation at 72°C for 30 sec; each sample was assayed in triplicate. A temperature range of 65–95°C was selected for drawing melting curves.

### Cell culture

Primary cultures of rat aortic vascular smooth muscle (VSM) cells, passage 2-10, were generously provided by Dr. Michael Crow of the National Institute of Aging. VSM cells were maintained in Dulbecco's modified Eagle's medium supplemented with 10% fetal bovine serum and gentamicin (50 μg/ml). Cultures were maintained at 37°C in a humidified atmosphere of 5% CO2, 95% air. Cells were exposed to hypoxia (1% O2, 5% CO2, balance N2) in a tightly sealed modular incubator chamber (Billups-Rothberg, Del Mar, CA) at 37°C. All experimentations were performed with confluent cultures.

### Cell transfection

HIF-1α plasmids and control vector were all obtained from Ambion (Ambion, USA). And then cell transfection was carried out using lipofectamine 2000 (Life Technologies, USA) according to manufacturer's instructions. Cells growing in 6-well plates were incubated with human siRNAs (100 nmol/L) for HIF-1α. Mock-transfection was performed using a negative control siRNA (Santa Cruz Biotechnology) as control. Cells were harvested at 48 h post transfection, washed and stored for future experiments. The knockdown efficiency was assessed using RT-PCR and western blot assay.

### Apoptosis assay

Cell apoptosis was analyzed by annexin V-FITC assay. Briefly, cells were stained with annexin V-FITC and propidium iodide using the ANNEXIN V-FITC Kit (Beckman) according to the manufacturer's protocol and subjected to flow cytometric analysis. Viable cells were not stained by annexin V or propidium iodide; early apoptotic cells were stained by annexin V but not propidium iodide whilst late apoptotic cells were stained by annexin V and propidium iodide.

### Cell counting kit-8 assay (CCK-8)

When the cells reached 90% confluence, they were then counted using a hemocytometer. After the cell concentration was adjusted to 2×105 cells/mL, these cells were added to 60 wells (100 μL per well) in the center of a 96-well plate, while an equal volume of PBS was added to the remaining surrounding wells. After labeling, the cell culture plate was placed in the incubator for 24 hours. This step was followed by serum-starvation with the same volume of serum-free medium for 24 hours, and the cells were then washed once with PBS. The cells were grouped and treated according to the above-described treatments (100 μL was added to each well). Twelve replicates were performed for each of the five treatment groups, and the cells were cultured for 24 h after treatment. A 10% CCK-8 solution was prepared by adding 1.2 mL of CCK-8 into 12 mL of DMEM. Treated cells were washed with PBS, and 100 μL of 10% CCK-8 was added to each well. After incubation for 3 h, the absorbance (OD) at 450 nm was measured using a microplate reader.

### TUNEL staining

The TUNEL reaction was performed with an *in situ* cell detection kit (Roche Applied Science, Indianapolis, IN, USA), according to the manufacturer's instruction, to detect the apoptosis of media cells. TUNEL-positive nuclei (stained brown) were counted by Motic Images Advanced 3.2 in 10 random fields (×200), and then averaged.

### Transwell migration assays

The cells were counted using a hemocytometer, and the concentration was adjusted to 7.5×104 cells/ml. After labeling, the cells were cultured for 24 h and then washed once with PBS. The un-migrated cells on the upper chamber surface were wiped with a cotton ball. The migrated cells were fixed with 4% paraformaldehyde for 30 min, stained with crystal violet for 20 min, and washed three times with PBS. The residual dye on both surfaces of the chamber was washed. After air-drying, the filter membrane was cut with a blade and observed under a microscope on a microslide. Cell counting was conducted for three randomly selected fields.

### Statistical analysis

Statistical analysis was performed using the SPSS statistical software program (Version 19.0; SPSS, Chicago, IL, USA). Student's two-tailed t test was used to compare data between two groups. One-way ANOVA and Dunnett's test were used to compare data between three or more groups. P < 0.05 was considered statistically significant.
